The article "Feature Importance Score-Based Functional Link Artificial Neural Networks for Breast Cancer Classification" was retracted in 2024. Reasons: signs of a paper mill; suspected computer-generated content; unreliable results or conclusions; concerns about the data.

# Feature Importance Score-Based Functional Link Artificial Neural Networks for Breast Cancer Classification

**DOI:** 10.1155/2022/2696916

**Published:** 2022-04-02

**Authors:** Shatakshi Singh, Sunil Kumar Jangir, Manish Kumar, Madhushi Verma, Sunil Kumar, Tarandeep Singh Walia, S. M. Mostafa Kamal

**Affiliations:** ^1^Dept. of Computer Science and Engineering, Mody University of Science and Technology, Sikar 332001, India; ^2^Wisflux Pvt. Ltd, Jaipur, Rajasthan, India; ^3^Dept. of Biomedical Engineering, Mody University of Science and Technology, Sikar 332001, India; ^4^School of Computer Science Engineering and Technology, Bennett University, Greater Noida 201310, India; ^5^School of Computer Science, University of Petroleum and Energy Studies, Dehradun 248001, India; ^6^School of Computer Application, Lovely Professional University, Phagwara, India; ^7^Department of Mathematics, Islamic University, Kushtia 7003, Bangladesh

## Abstract

Growth of malignant tumors in the breast results in breast cancer. It is a cause of death of many women across the world. As a part of treatment, a woman might have to go through painful surgery and chemotherapy that may further lead to severe side effects. However, it is possible to cure it if it is diagnosed in the initial stage. Recently, many researchers have leveraged machine learning (ML) techniques to classify breast cancer. However, these methods are computationally expensive and prone to the overfitting problem. A simple single-layer neural network, i.e., functional link artificial neural network (FLANN), is proposed to overcome this problem. Further, the F-score is used to reduce the issue of overfitting by selecting features having a higher significance level. In this paper, FLANN is proposed to classify breast cancer using Wisconsin Breast Cancer Dataset (WBCD) (with 699 samples) and Wisconsin Diagnostic Breast Cancer (WDBC) (with 569 samples) datasets. Experimental results reveal that the proposed models can diagnose breast cancer with higher performance. The proposed model can be used in the early breast cancer diagnosis with 99.41% accuracy.

## 1. Introduction

Cancer can spread in the whole body and accounts for the estimation of 9.6 million deaths worldwide, out of which 2.06 million deaths were caused due to breast cancer [1]. Similarly, breast cancer is caused by the growth of malignant tumors in the breast. It can be cured if it is diagnosed at an early stage. The World Health Organization (WHO) says that the survivability rate decreases from developed to developing countries due to inadequate diagnosis facilities [2].

In recent years, ML has majorly been applied in health informatics to predict various diseases as they can decrease the diagnosis time and find hidden relationships between complex datasets, which is indeed a tedious task for humans [3]. Various classification techniques such as SVM, KNN, logistic regression (LR), and NB have been used along with various supportive techniques like feature selection and feature extraction to reduce the error rate and overfitting [4]. However, if one algorithm is not efficient enough, then ensemble techniques are used to improve the accuracy and make the algorithm more effective [5].Chen et al. applied the rough set-support vector machine (RS-SVM) and divided datasets in 70%-30% and 50%-50% using a 5-fold cross-validation technique during experimentation [6]. Osman, A.H., has used a two-step SVM technique in which the first step is the clustering technique which is used to find the hidden pattern and SVM is used for classification [7]. As the application of AI and ML rise for the diagnosis of diseases, it can improve the efficiency and accuracy of the breast cancer diagnosis. Such an AI powered system could help to save lives by diagnosing cancer at an early stage and prevent the deaths in women due to breast cancer [8]. AI will not only help to make the process more accurate but also help the clinicians to speed up the diagnosis with the prescreening test [9]. This paper evaluates various researchers who have worked on WBCD and WDBC datasets to classify breast cancer and compare the accuracy, precision, recall, and specificity of classification techniques applied on these datasets to classify breast-cancer.

The article "Feature Importance Score-Based Functional Link Artificial Neural Networks for Breast Cancer Classification" was retracted in 2024. Reasons: signs of a paper mill; suspected computer-generated content; unreliable results or conclusions; concerns about the data.

Following are the significant contributions of this research article:

1. A novel functional link artificial neural network (FLANN)–based classifier is proposed to classify breast cancer with selected features. As per the authors' knowledge, functional link artificial neural network for the classification of breast cancer is first introduced and applied on two datasets with different features
2. Significant features have been selected based on the F-score for the classifier's training to reduce the complexity
3. The accuracy of the classifier is also examined based on selected breast cancer attributes
4. Different algorithms, including SVM, KNN, RF, NB, and MLP, have been implemented on WBCD and WDBC datasets, and their performance is compared with the proposed FLANN

The rest of the paper is arranged as follows: Related work is discussed in Section 2, highlighting some of the existing works of other researchers. In Section 3, various classification techniques implemented in this work and performance measurement techniques are discussed followed by the Results and Discussion presented in Section 4. Finally, the conclusion of this research paper is given.

The article "Feature Importance Score-Based Functional Link Artificial Neural Networks for Breast Cancer Classification" was retracted in 2024. Reasons: signs of a paper mill; suspected computer-generated content; unreliable results or conclusions; concerns about the data.

## 2. Related Work

Abonyi and Szeifert have examined supervised fuzzy clustering using 5 to 6 features and a 10-fold cross-validation technique and got the classification accuracy of 95.06% [8]. Othman and Yau have compared the performance of different algorithms including Bayes network, pruned tree, single conjunctive rule learner, radial basis function, and nearest neighbors algorithm using the WEKA data mining tool and achieved the highest accuracy of 89.71% from Bayes network [9]. Rong and Yuan have developed the SVM-KNN technique in which they applied KNN near hyperplane and SVM when the point is farther, achieving 98.06% accuracy [10]. Aruna and Nandakishore had compared NB, SVM, and decision tree using WEKA Tool and found SVM as the best with an accuracy of 96.99% [11]. Salama et al. presented a comparison of multilayer perceptron (MLP), Naive Bayes (NB), sequential minimal optimization (SMO), and KNN and used principal component analysis (PCA) for feature reduction, and then they obtained an accuracy of 97.1388% [12].

Gayathri and Sumanthi have presented the concept of relevance vector machine (RVM) and used the linear discriminant algorithm (LDA) [13] to reduce features to 4 and get the accuracy of 96% [14]. Shahnaz et al. compared NB, SVM, MLP, CNN, logistic regression, and KNN [15]. Li and Chen compared decision tree, SVM, random forest, LR, and NN models by dividing train and test set in 70%-30% and found that random forest is most suitable as it gave the highest accuracy 96.1%, highest area under the curve (AUC), and highest F-measure metric [16]. Adel S. Assiri et al. used a voting-based ensemble algorithm with the three best classifiers which are chosen based on their F3 score of 99.42% on the WBCD dataset [17]. T. Admassu optimized the KNN technique to optimize the Wisconsin Breast Cancer Dataset [18]. M. Zohaib et al. demonstrated that with feature selection based on chi-square, the optimal value for KNN for WBC and WBCD datasets is in the range 1-9 with the Manhattan or Canberra distance functions to measure the distance between points [19].

Md. Milo Islam et al. proposed a system utilizing SVM and KNN with a K-fold cross-validation method and suggested that SVM performs better on the WBCD dataset than the KNN algorithm with an accuracy of 98.57% and specificity of 95.5% [20]. Chaurasia V. et al. applied six different ML algorithms on WDBC with all the features and then reduced the features using statistical measures before applying the stacked classifiers to minimize the probability of misclassification in results [21]. In addition, various researchers have worked on different ML techniques to classify breast cancer types. It is found that the existing models suffer from the gradient vanishing [22–24], overfitting [25, 26], and data leakage [27, 28] kind of problems. Even development of generalized model [34,35] is still defined as an ill-posed problem.

The article "Feature Importance Score-Based Functional Link Artificial Neural Networks for Breast Cancer Classification" was retracted in 2024. Reasons: signs of a paper mill; suspected computer-generated content; unreliable results or conclusions; concerns about the data.

Table 1 presents the work of the various researchers who contributed to the same domain.

## 3. Methodology

Neural networks are often preferred for solving nonlinear problems [18]. FLANN is a high-order functional link–based single layer artificial neural network. There are no hidden layers in its architecture; therefore, it provides high convergence speed compared to other networks [19]. The structure of FLANN is given in Figure 1, where input features are expanded using nonlinear mathematical functions such as exponential, trigonometric, logarithmic, power, and Chebyshev functions. In the proposed methodology, features in the breast cancer dataset are expanded using trigonometric functions, depicted in Equation (2).

The breast cancer feature input is stored in a vector containing *n* different features which is given as

(1) $$\begin{array}{c} X={\left[x_{1}x_{2}\cdots x_{n}\right]}^{T}, \end{array}$$

where *X* can be further expanded using trigonometric functions as

(2) $$\begin{array}{c} X={\left[x_{1}\cos\left(\pi x_{1}\right)\sin\left(\pi x_{1}\right)\cdots \cos\left(2\pi x_{1}\right)\cdots x_{2}\cos\left(\pi x_{2}\right)\;\sin\left(\pi x_{2}\right)\cdots \cos\left(2\pi x_{2}\right)\;\sin\left(2\pi x_{2}\right)\cdots x_{1}x_{2}\right]}^{T}. \end{array}$$

After expansion of the input feature, weights will be initialized randomly, and it is given as

(3) $$\begin{array}{c} W={\left[w_{0}w_{1}\;w_{2}\cdots w_{n-1}\right]}^{T}. \end{array}$$

The weighted sum of input and bias will provide output *Y*^(*j*)^.

(4) $$\begin{array}{c} Y^{\left(j\right)}=\overset{n-1}{\underset{k=0}{\sum }}x_{k}^{\left(j\right)}W_{k}. \end{array}$$

*Y* ^(*j*)^ is then passed through a nonlinear hyperbolic logarithmic activation function as

(5) $$\begin{array}{c} y^{\left(j\right)}=\frac{1}{2}\;\log_{e}\frac{1+Y^{\left(j\right)}}{1-Y^{\left(j\right)}}. \end{array}$$

Network error of FLANN can be computed by

(6) $$\begin{array}{c} \varepsilon_{j}\left(n\right)=d^{\left(j\right)}-y^{\left(j\right)}. \end{array}$$

The weights of the FLANN network is updated by applying the backpropagation algorithm, given as

(7) $$\begin{array}{c} w_{ij}^{\left(l\right)}\left(n+1\right)=w_{ij}^{\left(l\right)}\left(n\right)+\alpha {∆}_{ij}\left(n\right), \end{array}$$

where *w*_*ij*_^(*l*)^(*n* + 1) is an updated weight, similarly, *w*_*ij*_^(*l*)^(*n*) is the old weight, and *α* denotes the learning rate.

∆_*ij*_(*n*) = *δ*_*i*_^(*l* + 1)^*x*_*j*_^(*l*)^, *l* = *L* − 1, *L* − 2, ⋯, 0, where *L* denotes current layer.

*δ*_*i*_^(*p*)^ = *ε*_*j*_(*n*)*g*′(*S*_*i*_^(*p*)^), for the output layer.

 = [∑_*k*=1_^*N*_*p*+1_^*δ*_*k*_^(*p* + 1)^*w*_*ki*_^(*p*)^(*n*)]*g*′(*S*_*i*_^(*p*)^), for the other layers.

The article "Feature Importance Score-Based Functional Link Artificial Neural Networks for Breast Cancer Classification" was retracted in 2024. Reasons: signs of a paper mill; suspected computer-generated content; unreliable results or conclusions; concerns about the data.

Table 2 shows the properties of SVM, MLP, DT, KNN, and NB, and these properties can be used to get better accuracy and will help in selecting an algorithm according to the need. Apart from accuracy, researchers have worked on various other metrics to evaluate the performance of the different ML algorithms. Various quality metrics such as confusion matrix, precision, specificity, accuracy, and recall are used to measure implemented ML algorithms' performance [31]. The confusion matrix represents the data graphically, and values in the matrix are represented using colors. They include the information about the actual and classified output of the input data points. The abovementioned metrics can be mathematically represented as

(8) $$\begin{array}{c} \text{Accuracy}=\frac{\;TP+TN}{N},\\ \text{Precision}=\frac{TP}{TP+FP},\\ \text{Recall}=\frac{TP}{TP+FN},\\ \text{Specificity}=\frac{TN}{\;TN+FP}, \end{array}$$

where TP represents true positive results, FP is the false positives, TN is the number of true negative results, and FN denotes the false negatives in the output. Equations (8) presents the mathematical form of performance measurement criteria, and Table 3 shows the confusion matrix components which can be used to evaluate any algorithm.

## 4. Results and Discussion

The simulation work was done in the Google Colaboratory (Google Colab). It is a cloud-based Jupyter Notebook that uses Python version 3.6 platform. It provides decent computation power, 12.72 GB Random Access Memory (RAM) and 68 GB disk storage. In this study, various machine learning-based classification algorithms have been used to train the models using two different breast cancer datasets: Wisconsin Breast Cancer Dataset (WBCD) [32] and Wisconsin Diagnostic Breast Cancer Dataset (WDBC) [33]. Their performance has been compared with FLANN considering the different number of features.

WBCD contains 11 columns, out of which the first column is “sample id,” which is not relevant, and the last column of the dataset contains the output, which exhibits whether the tumor is benign or malignant. In this dataset, there are 699 samples, out of which 458 (65.5%) are benign and 341 (35.5%) are malignant. In WBCD (original), 16 values are missing, which have been replaced with the mean value.

The F-score of each feature is shown in Figure 2 to determine the significance level of each feature, using which we found that feature numbers f5, f0, f7, and f3 play a significant role in classifying breast cancer. F-score can be computed with the help of confusion matrix for every feature. The feature importance is calculated for every decision tree by the amount that each attribute split point improves the performance measure, weighted by the number of observations the node is responsible for.

The article "Feature Importance Score-Based Functional Link Artificial Neural Networks for Breast Cancer Classification" was retracted in 2024. Reasons: signs of a paper mill; suspected computer-generated content; unreliable results or conclusions; concerns about the data.

The FLANN is compared with other classification techniques such as NB, SVM, RF, KNN, and MLP. The comparison study is depicted in Table 4. This table also gives the accuracy level on various features level and is selected by applying the F-score method.

The experimental results of Table 4 reveal that all the algorithms perform well, particularly with three features, i.e., *Bare Nuclei*, *Clump Thickness* and *Normal Nucleoli*. SVM outperformed the other ML techniques, and accuracy reached 97.8%, whereas 97.14% accuracy was obtained using FLANN. The above result demonstrates that the result mainly relies upon the significant features only, thereby eliminating redundant attributes for the training of the ML models. Furthermore, it will not only help to reduce computational complexity but also in expediting the learning process of ML techniques. Finally, the confusion matrix of classification using SVM with three features is presented in Figure 3.

This confusion matrix provides different quality metric data such as precision (0.976), recall (0.9888) and specificity (0.964). Likewise, MLP consists of multiple perceptron in each layer and is applied to the WBCD dataset. The batch size is taken as 16, and categorical cross-entropy is used to calculate the loss. Also, Adam's optimizer is a learning algorithm. The accuracy obtained by the MLP on only two features is 94.28%, with three features is 96.85% and with five features is 95.28%. The loss and accuracy after each epoch can be depicted using the graphs Figures 4 and 5.

The above graphs demonstrate the accuracy of the training and a testing dataset. Initially, the graph increases exponentially and then increases, and after a few epochs, the accuracy becomes saturated. The model's accuracy may change with the learning rate and other ML network parameters. Similarly, the model loss is inversely proportional to the accuracy. Hence the graph decreases exponentially and is then saturated with the epoch. Since WBCD (Original) has only ten features and only one value ranging from 1-10 is considered, another dataset, i.e., WDBC having more features, was considered for the experiments.

Similarly, in WDBC, there are ten features followed by the mean of values, standard error and the maximum value of the mean of the largest three values of features for each property, making it a total of 30 features. The input values of the selected features are obtained using the digitized image of the fine needle aspirant technique, and all feature values are recoded with up to four significant digits. There are no missing values in the dataset. This dataset contains 569 samples, of which 357(62.74%) are benign and 212(37.25%) malignant. This F-score of each feature is shown in Figure 6.

The article "Feature Importance Score-Based Functional Link Artificial Neural Networks for Breast Cancer Classification" was retracted in 2024. Reasons: signs of a paper mill; suspected computer-generated content; unreliable results or conclusions; concerns about the data.

Using Figure 6 it is found that f21, f23, f13, f27, f1, f26, f7, f24, f4 and f15 play a major role in classifying breast cancer. Table.  5 shows the result of the experiment of different algorithms with various numbers of features.

SVM and Naive Bayes work better with six major features, FLANN with 11 features, and random forest with all the features.

From Figure 7, we can calculate the precision (97.2%), recall (100%), and specificity (95.34%). Apart from these machine learning techniques, MLP also performs well in classifying the tumor, and data are trained in the batch size of 16. The categorical cross-entropy and Adam's optimizer were calculated to improve the accuracy level. After each forward propagation loss is calculated, the weight parameters are changed to reduce the loss and increase accuracy. The accuracy obtained when using six features is 96.49%, with 11 features 96.49%, and the highest accuracy of 97.28% was obtained when all the features were considered. Figures 8 and 9 show the accuracy and loss after each epoch when all the features are used.

From both the above graphs, it can be concluded that loss and accuracy have an inverse relation. In the initial epochs, accuracy increases rapidly, and loss decreases, and after that rate of change of both accuracy and loss decreases, and after a few epochs, they change negligibly. Hence, the training is stopped without further delay. From Table 4 and Table 5, it can be concluded that for most machine learning techniques, better results are obtained for WDBC using the same classification algorithm, but WBCD did better when FLANN was used and achieved accuracy 99.41%, which is the best among all.

It can be observed that ML algorithms like NB, KNN, and SVM were able to achieve the accuracy obtained by FLANN. These algorithms have certain demerits which make it infeasible to use them for diagnosis. Naive Bayes has a strong assumption that is unrealistic for real-world data that all the input features are independent. KNN, despite of being a machine learning algorithm, cannot be used to train a model. There is no training involved when we use KNN. At the time of query, the *k* data points close to the query point are considered, and final output is decided. Hence, all the data need to be stored in the system and has to be accessed for each single query. SVM aso required the training data to be loaded in memory at once. This makes the algorithm computationally very expensive and unrealistic for the real-time implementation.

The article "Feature Importance Score-Based Functional Link Artificial Neural Networks for Breast Cancer Classification" was retracted in 2024. Reasons: signs of a paper mill; suspected computer-generated content; unreliable results or conclusions; concerns about the data.

## 5. Conclusions

This paper presents the study based on machine learning algorithms to diagnose breast cancer using physiological measures. WBCD and WDBC datasets are used for the study. The feature selection techniques are applied to select the most significant features in the dataset. Further, the accuracy is compared based on feature selection. To avoid the overfitting issue, this paper presents a FLANN algorithm for classification on two datasets WBCD and WDBC. This algorithm is computationally effective, more accurate, and converges faster than other algorithms because it has no hidden layer. The experimental studies conclude that an accuracy of 99.41% is achieved using the proposed FLANN with all features on the WDBC dataset. WDBC dataset is better as it considers dispersion factors like the standard deviation of the features that are important in breast cancer classification. In the future, X-ray images can be used to classify cancers using deep learning. However, X-ray is more feasible than the fine needle aspirant technique and uses the regional dataset to address a specific cancer problem.

## Figures and Tables

**Figure 1:** Architecture of functional link artificial neural network.

**Figure 2:** Feature importance score of all the features in dataset.

**Figure 3:** Confusion Matrix of SVM with three features.

**Figure 4:** Model Accuracy of MLP.

**Figure 5:** Model-Loss after each epoch.

**Figure 6:** F-Score of all the features.

**Figure 7:** Confusion matrix of SVM with six features.

**Figure 8:** Accuracy of a model after each epoch.

**Figure 9:** Loss of model after each epoch.

**Table 1:** Research work available in literature for the classification of breast cancer using artificial intelligence (AI).

Study	Year	Algorithm	Accuracy
Pene-Rayes and Sipper [1]	1999	Fuzzy-GA	97.36%
Abbass [2]	2002	MPANN	98.1%
Guo and Nandi [10]	2006	MLP	97.89%
Übeyli, E.D. [11]	2007	PNN (probabilistic neural network)	98.15%
Subashini et al. [12]	2009	RBFNN	96.57%
Fatima and Amine [6]	2012	Hybrid neuro-fuzzy	98.25%
Manning and Walsh [7]	2013	CGPANN	96%
Zeng et al. [13]	2014	SVM-KNN	97.38%
Banerjee et al. [14]	2017	Ensemble	95.6%
Amrane et al. [15]	2018	KNN	97.51%
Alwidian et al. [16]	2018	WCBA	97.74%
Bayrak et al. [17]	2019	ANN	95.42%

**Table 2:** Advantages and disadvantages of various ML algorithms [20–37].

Technique	Advantage	Disadvantage
SVM	It allows the generation of nonlinear boundaries	Choice of kernel
MLP	Ability to learn on its own	Complexity is high
DT	Independence of variables is not required. Easy to understand	High probability of overfitting
KNN	Training time is negligible	Does not work well with large dataset
NB	Training time remains constant irrespective of size	Features should be independent of each other

The article "Feature Importance Score-Based Functional Link Artificial Neural Networks for Breast Cancer Classification" was retracted in 2024. Reasons: signs of a paper mill; suspected computer-generated content; unreliable results or conclusions; concerns about the data.

**Table 3:** Confusion matrix.

	Predicted yes	Predicted no
Actual yes	TP	FN
Actual no	FP	TN

**Table 4:** Accuracy of classifiers on WBCD.

Features	Accuracy		
	5	3	2
Techniques			
SVM	97.14%	97.8%	95.7%
Naïve Bayes	96.42%	97.14%	97.14%
Random Forest	97.14%	97.14%	93.57%
KNN	95.71%	95.71%	97.8%
MLP	95.28%,	96.85%	94.28%.
FLANN	97.14%	96.88%	96.76%

**Table 5:** Results of Machine Learning Techniques on WDBC.

Technique	Accuracy when the number of features are		
	6	11	30
SVM	98.24%	97.36%	98.24%
KNN	95.61%	96.49%	96.49%
Random forest	96.49%	92.98%	97.14%
Naive Bayes	97.36%	96.49%	96.49%
MLP	96.49%	96.49%	97.28%
FLANN	95.57%	97.45%	99.41%

## Data Availability

The data used is freely available at https://archive.ics.uci.edu/ml/datasets/breast+cancer+wisconsin+(original) and https://archive.ics.uci.edu/ml/datasets/breast+cancer+wisconsin+(diagnostic).
